# Integrative Bioinformatics Analysis Reveals That miR-524-5p/MEF2C Regulates Bone Metastasis in Prostate Cancer and Breast Cancer

**DOI:** 10.1155/2022/5211329

**Published:** 2022-09-10

**Authors:** QingHua Tian, YingYing Lu, BiCong Yan, ChunGen Wu

**Affiliations:** Department of Diagnostic and Interventional Radiology, Shanghai Jiao Tong University Affiliated Sixth People's Hospital, Shanghai, China

## Abstract

Bone metastases are highly prevalent in patients with advanced prostate cancer and breast cancer and have a serious impact on the survival time and quality of life of these patients. It has been reported that microRNAs (miRNAs) are expressed abnormally in different types of cancer and metastases. However, it remains unknown whether the underlying miRNAs are associated with prostate and breast cancer bone metastasis. Differentially expressed miRNAs (DE-miRNAs) and their potential targets in the metastatic process were identified by bioinformatics analysis. Additionally, qPCR confirmed that the miR-524-5p expression was downregulated in prostate and breast cancer cells. The overexpression of miR-524-5p restrained cell proliferation, invasion, and metastasis in prostate and breast cancer cells. Meanwhile, miR-524-5p could target and inhibit the expression of MEF2C, which was verified by a luciferase assay. In conclusion, our data strongly suggest that downregulation of miR-524-5p appears to be a precocious event in prostate and breast cancer, and the miR-524-5p/MEF2C axis plays a novel role in bone metastases from prostate and breast cancers.

## 1. Introduction

Prostate cancer and breast cancer are the two most common invasive cancers in men and women, respectively. Although these two cancers arise from different organs, they are typically hormone-dependent and have an underlying biological mechanism in common [1]. As cancer is a metastatic disease, hormone therapy plays an essential role in receptor-positive breast and prostate cancer. However, although hormone therapy initially has an effect on the inhibition of breast and prostate tumours, bone metastasis is still a problem for 70% of metastatic prostate and breast cancer patients [2], showing a poor prognosis. In addition, prostate cancer and breast cancer are malignancies that are destined to become metastatic if screening has been unable to identify them at an early stage before symptoms appear [3], causing a serious threat to patients' lives.

Bone is the tissue most susceptible to metastasis in prostate cancer [4] and breast cancer [5]. Once cancer has metastasized to the bones, and numerous skeletal-related events (SREs), such as fracture, intractable pain, bone marrow aplasia, nerve compression syndrome, and spinal cord compression, occur [6], which can rarely be cured and result in significant morbidity in patients with prostate cancer and breast cancer. Despite its morbidity, bone metastasis is one of the most intriguing and complex biological processes of all oncogenic processes and consists of the three key steps of seeding, dormancy, and outgrowth [7]. All of the processes involved in metastasis and interaction with host cells can be targeted to treat bone metastasis and tumor progression in prostate cancer and breast cancer.

MicroRNAs (miRNAs or miRs-), which are 21-25 nucleotides long, are single-stranded noncoding RNAs that are evolutionarily conserved and endogenously produced. miRNAs play an essential role in targeting the 3′ untranslated region (3′ UTR) of mRNAs, mainly to repress their expression [8]. Over the past several years, many miRNAs have been found and characterized in the pathogenesis of many human malignancies, including critical chemokines and cytokines in the bone metastasis microenvironment [9, 10]. For example, it was reported that miR-124 could inhibit bone metastasis by inhibiting interleukin-11 in breast cancer [11]. miR-133a-3p represses bone metastasis of prostate cancer [12]. In addition, the occurrence and development of many kinds of cancer, such as colon cancer [13], melanoma [14], gastric cancer [15], osteosarcoma [16], ameloblastoma [17], and particularly breast cancer [18], are highly associated with the abnormal expression of miRNAs. Jin et al. identified miR-524-5p as a tumor suppressor. Moreover, miR-524-5p inhibited cell migration, invasion, and epithelial–mesenchymal transition and progression in breast cancer [18]. However, little is known about its function in bone metastases of prostate and breast cancer.

Here, for the first time, we revealed the role of cancer cell-derived miR-524-5p in bone metastases of prostate cancer and breast cancer. Perturbation of the miR-524-5p/MEF2C regulatory axis contributes to bone metastasis in prostate cancer and breast cancer. These results might provide novel therapeutic and diagnostic targets for bone metastases of breast cancer and prostate cancer.

## 2. Materials and Methods

### 2.1. Download of mRNA and miRNA Expression Profiles

The expression of genes and miRNAs between patients with primary prostate and breast cancer with bone metastatic prostate and breast cancer was compared. The Gene Expression Omnibus (GEO) database (https://www.ncbi.nlm.nih.gov/geo/) was employed to obtain the gene expression profiles and the miRNA expression profile. One dataset, GSE32269, deposited by Cai et al. [19], contains 22 primary prostate cancer (hormone-dependent) versus 29 metastatic prostate cancer samples. Another dataset, GSE137842, was submitted by Lefley et al. [20] and contains 3 primary breast cancer and 3 breast cancer bone metastasis samples. These two datasets were acquired from the Affymetrix Human Genome U133 Plus 2.0 Array. The miRNA microarray dataset GSE26964 [21] was composed of 6 primary prostate cancer samples and 7 prostate cancer bone metastatic samples (platform: Capitalbio mammal microRNA V3.0).

### 2.2. Identification of Differentially Expressed miRNAs and mRNAs

Herein, the mRNA and miRNA expression profile data preprocessing mainly consists of background correction, quantile normalization, and probe summarization [22]. Then, limma package in bioconductor was used to extract differentially expressed miRNAs (DE-miRNAs) and differentially expressed genes (DEGs) [23] following criterion *P* value <0.05 and   | log_2_foldchange | >1.

### 2.3. GO and KEGG Pathway Annotation

The online tool of Database for Annotation and Visualization and Integrated Discovery (DAVID) was used to perform Gene Ontology (GO) and Kyoto Encyclopedia of Genes and Genomes (KEGG) functional enrichment of the identified common DEGs and DE-miRNAs [24, 25]. GO analysis was conducted for the cellular component (CC), biological process (BP), molecular function (MF) categories [26], and KEGG pathway enrichment analysis for the selected genes [27]. All parameters were set as default, and *P* value <0.01 was considered significant.

### 2.4. Construction of the mRNA–miRNA Regulation Network

miRBase, TargetScan (http://www.targetscan.org/vert_71/), miTarBase, and miRWalk databases were used to identify the number of miRNA-regulated target gene pairs. The threshold of the correlation coefficient was set as -0.3, and the significance *P* value was set as 0.05. The pairs supported by two or more databases were further processed and retained. Regulatory network visualization for the regulatory relationship between miRNA-mRNA was conducted using Cytoscape [28].

### 2.5. PPI Network and Hub Gene Analysis

The interaction of the DEGs was detected using the Search Tool for the Retrieval of Interacting Genes (STRING) database, with confidence scores > 0.7. Cytoscape was used to visualize the PPI network. Hub genes and screen modules of the PPI network were identified using the CytoHubba plug-in and Molecular Complex Detection (MCODE) plug-in, of which all of the parameters were left as the defaults. Metascape was used to analyze the genes in modules.

### 2.6. Cell Culture

The DU145 and LNCAP cell lines of human prostate cancer and MCF7 of breast cancer were obtained from COWELDGEN SCIENTIFIC (Coweldgen Scientific Co., Ltd., Shanghai, China). DU145 and MCF-7cells were cultured in MEM (Invitrogen, USA) supplemented with 10% FBS (Invitrogen, USA). LNCAP was cultured in RPMI 1640 medium (Invitrogen, USA) with 10% FBS. All medium were supplemented with penicillin (100 U/ml) and streptomycin (100 mg/ml) (Biosharp, China). All cells were cultured at 5% CO_2_ and 37°C humidified atmosphere.

### 2.7. Cell Transfection

Transfection was conducted when the cell density reached 70-80% in six-well plates. miR-524-5p mimics and negative control (NC) were designed and synthesized by GenePharma (Shanghai, China). miR-524-5p mimics or NC (50 nM) was transfected into cells using Lipofectamine 3000 (Invitrogen, USA) following the manufacturer's instructions.

### 2.8. RNA Extraction and qPCR Analyses

Total RNA was extracted from cell lines with TRIzol Reagent (Invitrogen, USA) following the manufacturer's instructions. In details, total RNA (2.0 *μ*g) was reverse transcribed using the PrimeScript TM RT reagent Kit (Takara, Japan) following the manufacturer's instructions. cDNA was amplified and quantified on the LightCycler® 96 system (Roche, Switzerland) usingSYBR® Premix Ex Taq™ II (Takara, Japan). miRcute Plus miRNA First-Strand cDNA Kit (TianGen Biotech, Beijing, China) and SYBR Green (Takara, Japan) were used to quantify mature miRNA levels. 2^-*ΔΔ*Ct^ was calculated to represent the relative fold expressions. The primers are shown in Table 1.

### 2.9. Western Blot

Total protein was extracted from cell lysate using PMSF. Then, protein sample was quantified by bicinchoninic acid (BCA), separated by SDS-PAGE gel electrophoresis, and blocked with 5% skim milk. After that, membranes were incubated with the specific primary antibody at 4°C overnight. Membranes were washed three times using TBST and incubated with the corresponding HRP-conjugated secondary antibody for 2 h at room temperature. Enhanced chemiluminescence (PerkinElmer) was used to expose membranes after washing three times. Western blots were quantified by densitometry using ImageJ.

### 2.10. Dual-Luciferase Reporter Gene Assay

The 3′ UTR sequence of MEF2C containing wild-type or mutant binding sites was cloned into the pmirGLO luciferase vector. Then, the MEF2C 3′ UTR WT or MUT and miR-524-5p mimics or negative control were cotransfected using Lipofectamine 3000. After 72 h, the cell lysate was centrifuged at 12,000 rpm for 5 min to perform the Dual-Lumi Luciferase Assay (Beyotime Biotechnology, Shanghai, China). Luciferase activity was measured by an EnVision Multifunctional Microplate Reader (PerkinElmer, Germany).

### 2.11. Cell Counting Kit-8 (CCK-8) Assay

A 100 *μ*L cell suspension (1 × 10^4^ cells) was placed in each well of a 96-well plate. Ten microliters of CCK-8 reagent (Beyotime Biotechnology, Shanghai, China) was added at 6 h, 24 h, 48 h, 72 h, and 96 h. Then, the cells were cultured for 2 h, and the absorbance value was detected at a wavelength of 450 nm by a microplate reader (SpectraMax M5; Molecular Devices, USA).

### 2.12. Transwell Assay

A cell suspension (1 × 10^5^ cells/ml) was prepared with serum-free medium. Then, 100 *μ*L suspension was added to the chamber, and 600 *μ*L of complete medium was supplied to the basolateral chamber, which was incubated overnight. Subsequently, unpenetrating cells above the chamber were removed, the chamber was fixed in 4% paraformaldehyde for 30 min and then dyed with 1% crystal violet for 10-15 min, and five randomly selected fields were captured using an inverted microscope (Olympus, Tokyo, Japan).

### 2.13. In Vitro 3D Model of Prostate and Breast Cancer Metastasis

The animal experiments performed in this study were approved by the Institutional Animal Care and Use Committee of ShangHai Sixth People's Hospital. To imitate the bone metastasis microenvironment in vivo, neonatal CD-1 mice were used to build an in vitro 3D model. In detail, after CD-1 mice were sacrificed, their calvarial bone was separated under sterile conditions and cut in the occipital lobe to produce an arch structure [29]. Then, calvarial bones were washed with PBS and cocultured with DU145 cells or MCF7 cells and DU145 cells or MCF7 cells transfected with miR-524-5p mimics in a 48-well plate (5 × 10^5^ cells). Cranium bones without culturing with cells were used as a negative control. The crystal violet staining experiment was performed after incubation at 37°C for 4 days. In brief, the bone fragments were removed, fixed with 95% alcohol for 10 min, washed with PBS 3 times, and stained with 5 mg/ml crystal violet for 15 min. The stained bone slices were washed with PBS 3 times and observed under an inverted microscope. Each bone slice was randomly taken from 3 different fields to count the adhered cells [30, 31].

### 2.14. Statistical Processing

SPSS software (22.0, US) was utilized for statistical analysis. All data were represented as mean ± SD. Statistical differences were determined by a one or two-sided Student's *t*-tests ort wo-way ANOVAs. A *P* value <0.05 was considered statistically significant.

## 3. Results

### 3.1. Identification of DE-miRNAs and DEGs

A total of 1555 DEGs were obtained from breast cancer gene expression profiles of GSE137842, of which 625 DEGs were overexpressed and 930 DEGs were downregulated in breast cancer bone metastasis samples compared to primary breast cancer samples. Volcano plots were generated to visualize all the DEGs (Figures 1(a) and 1(b)). A total of 833 DEGs were identified from prostate cancer gene expression profiles of GSE32269, of which 522 were upregulated and 311 were downregulated in prostate cancer bone metastasis samples compared to primary prostate cancer samples. Volcano plots were generated to visualize all the DEGs (Figures 1(c) and 1(d)). A total of 88 DE-miRNAs were obtained from prostate cancer miRNA expression profiles of GSE26964, of which 11 were upregulated and 77 were downregulated in prostate cancer bone metastatic samples compared to primary prostate cancer samples. Volcano plots were generated to visualize all DE-miRNAs (Figures 1(e) and 1(f)). We overlapped the DEGs (mRNA) screened in the prostate cancer bone metastasis dataset and breast cancer bone metastasis and identified 17 genes that were upregulated and 20 that were downregulated (Figures 1(g) and 1(h)).

### 3.2. Pathway and Process Enrichment Analysis of DEGs

For the selected common DEGs, pathway and process enrichment analyses were conducted through GO processes and KEGG pathways [32]. The representative top 15 clusters from the 3 categories are shown in Figure 2(a). The terms enriched in the biological process (BP) category included cardiac tissue and animal organ development, embryonic organ morphogenesis, cardiac muscle cell differentiation, bone development, and bone morphogenesis. The molecular function category demonstrated enrichment in factors involved in the extracellular exosome, collagen-containing extracellular matrix, cell-substrate adherens junction, and focal adhesion. In addition, the GO cell component category showed enrichment in cadherin binding, ribonuclease activity, retinoid binding, DNA binding, enhancer binding, and aminopeptidase activity.

The results from KEGG pathway enrichment analysis demonstrated that common DEGs were significantly involved in transcriptional misregulation in cancer, parathyroid hormone synthesis secretion and action, regulating pluripotency of stem cells, MAPK signaling, Ras signaling pathways, EGFR tyrosine kinase inhibitor resistance, prostate cancer, viral protein interaction with cytokine and cytokine receptor, FoxO adhesion molecules, gastric cancer, proteoglycans in cancer, and endocytosis (Figure 2(b)).

### 3.3. Construction of the mRNA–miRNA Regulation Network and PPI Network

Three target prediction databases were employed to identify the target genes of selected DE-miRNAs. In total, 37 miRNAs were identified for 88 DE-miRNAs, which had different expression levels between patients with primary prostate cancer and patients with prostate cancer bone metastasis. In addition, 13 of the target genes (MEF2C, ZC3H7B, HOXB7, MAFB, GART, CD163, RAPGEF5, DHX9, MXRA5, MMP16, GJA1, PRKCA, ASPN) were upregulated, and one was downregulated. Thirty-seven DE-miRNAs and 14 target genes were identified in the miRNA–mRNA regulatory network, as shown in Figure 3(a). Among those DEGs, MEF2C showed the extremely high expression in patients with bone metastatic prostate and breast cancer (Figure 3(b)). Notably, MEF2C was one of the targets of miR-524-5p.

PPI networks were constructed through the string database from 13 proteins (confidence level of 0.4) consisting of 13 nodes and 14 edges for the DEGs in bone metastasis. The PPI network analysis showed that MEF2C, FGFR2, IGF1, and NCAM1 were hub genes (Figure 3(c)).

### 3.4. miR-524-5p Overexpression Restored Cell Proliferation and Invasion in Prostate and Breast Cancer

miR-524-5p was found to be one of the most significantly downregulated miRNAs in prostate and breast cancer with bone metastasis (Figures 3(a) and 3(b)). To further validate this result, the expression of miR-524-5p in the human prostate cancer cell lines DU145 and LNCAP and breast cancer cell line MCF7 was measured. qPCR showed that the expression of miR-524-5p was lower in MCF7 and DU145 cell lines than in LNCAP (Figure 4(a)).

To explore the biological function of miR-524-5p, miR-524-5p mimics were transfected into DU145 and MCF7 cell lines. The expression of miR-524-5p in DU145 and MCF7 cells was significantly increased in transfected cells (Figure 4(b)). In the CCK-8 assay, the cell proliferation ability of DU145 and MCF7cells was inhibited by miR-524-5p mimics (Figure 4(c)). In the transwell assay, miR-524-5p mimics inhibited the migration ability of DU145 and MCF7 cells (Figure 4(d)).

### 3.5. miR-524-5p Specifically Targets MEF2C

MEF2C, a transcription factor, has been proposed as a new player in breast cancer brain metastasis development [33]. In contrast to miR-524-5p, MEF2C was upregulated in prostate and breast cancer with bone metastasis, and the MEF2C gene was predicted to be a target for miR-631, miR-524-5p, miR-330-3p, and miR-346 (Figure 3(a)). qPCR results showed that MEF2C mRNA significantly decreased in cells transfected with miR-524-5p mimics compared with the NC group (Figure 5(a)), and Western blotting demonstrated that the MEF2C protein was also dramatically decreased (Figure 5(b)). The data indicated that MEF2C is most likely the target of miR-524-5p.

TargetScan predicted that there were binding sites of miR-524-5p in the 3′ UTR of MEF2C at bases 130-136 (site 1) and 904-910 (site 2) (Figure 5(c)). To further confirm the inference that miR-524-5p targeted MEF2C, a luciferase reporter assay was conducted. For site 1, luciferase activities decreased in the cells cotransfected with wild-type MEF2C and miR-524-5p mimics compared with those in the NC group. However, there were no differences in the luciferase activities compared with their control group after cotransfection with MEF2C mutation (mut) and miR-524-5p mimics. For site 2, there was less change in the luciferase activities compared with those in their control group after cells were cotransfected with wild-type MEF2C and miR-524-5p mimics (Figure 5(d)). Therefore, MEF2C could be targeted by miR-524-5p through binding to both sites.

### 3.6. Effect of miR-524-5p on an In Vitro 3D Model of Prostate or Breast Cancer Bone Metastasis

Generally, the calvarial bone tissue was smooth and flat. However, in the model group cultured with DU145 or MCF7 cells, many DU145 or MCF7 cells obviously grew on the surface of calvarial bone. The number of DU145 or MCF7 cells on the calvarial bone was measured through crystal violet staining. The miR-524-5p mimics inhibited the growth of DU145 or MCF7 cells on the surface of the calvarial bone tissue (Figures 6(a) and 6(b)), which proved that the calvarial bone had strong adhesion to tumor cells. The adhered tumor cells caused damage to the calvarial bone in the coculture group. However, the overexpression of miR-524-5p repressed the adhesion and metastasis of tumor cells to bone tissue.

## 4. Discussion

As we described previously, bone is the most preferential metastatic site for prostate and breast cancer. Bone metastasis for prostate and breast cancer is a multistep process including tumor cell dissemination into the circulation, homing to the bone, and proliferation in bone tissue. A complicated network of molecular events plays an essential role in the development of bone metastasis. However, the underlying mechanism is not fully understood. In this study, a comprehensive genetic interaction network was established to explore the role of potential miRNAs, particularly miR-524-5p and its target MEF2C. We found that MEF2C was upregulated in bone metastasis development and regulated by miR-524-5p. These findings provide new insights into the altered miRNAs serving as potential biomarkers and MEF2C as a potential target for preventing or breaking prostate and breast cancer metastasis.

Several lines of literature have reported that miRNAs play a key role in cancer progression and metastasis. We found 11 downregulated miRNAs, including miR-524-5p, miR-330-3p, and miR-346, and 77 upregulated miRNAs, such as miR-564, miR-602, and miR-129-5p, when searching for miRNAs with aberrant expression in prostate metastasis. Overexpressed miRNAs in various tumors have been found to be oncogenic miRNAs [34–37]. Other miRNAs with decreased expression are predicted to be tumor suppressors [38–40]. Among those miRNAs, as revealed by target prediction, miR-524-5p emerged as the most promising molecule and was reported to be involved in various cancers through different mechanisms. It has been predicted that miR-524-5p plays a tumor suppressor role in multiple types of cancers. Several studies have reported that miR-524-5p was downregulated in tumors, including glioma [41], colon cancer cells [13], gastric cancer [15], and papillary thyroid carcinoma [42], which can inhibit tumor proliferation and metastasis. In breast cancer, Jin et al. found that miR-524-5p inhibited the progression of migration, invasion, and epithelial–mesenchymal transition by targeting FSTL1 [18]. Consistent with Jin et al.'s result, our study confirmed that miR-524-5p was downregulated in prostate cancer bone metastasis compared to its expression in primary prostate cancer, and that the expression of miR-524-5p inhibited cell proliferation and invasion ability. The contradictions in previous reports may have arisen because a single miRNA can regulate various genes and functions or influence the expression of multiple factors in different cellular contexts [43].

The myocyte enhancer factor 2 (MEF2) protein family includes MEF2A, MEF2B, MEF2C, and MEF2D. MEF2C is widely expressed in muscle, neuronal, chondroid, immune, and endothelial cells [44]. In addition, MEF2C has close connections with uncontrolled cancer cell proliferation and enhanced invasion [45]. Regarding cancer metastasis, a recent study reported that MEF2C was consistently expressed in breast cancer brain metastases, and that its nuclear translocation was related to brain metastatic disease severity via VEGFR-2 and *β*-catenin signaling [46]. MEF2C was predicted to be regulated by miR-802-5p and miR-194-5p in brain metastases of breast cancer, which indicates that MEF2C plays a role in tumor metastasis. In this study, we found that MEF2C is upregulated in prostate and breast cancer bone metastasis. MEF2C was regulated by miR-524-5p, which was confirmed by luciferase assays and in vitro experiments. The absence of miR-524-5p in primary cancer tissue may promote bone metastasis through the upregulation of MEF2C. However, the specific downstream mechanism involved needs to be further investigated. Collectively, downregulation of miR-524-5p appears to be a precocious event in prostate and breast cancer, and MEF2C serves as a new player in prostate and cancer bone metastasis development.

## Figures and Tables

**Figure 1:** Identification of DE-miRNAs and DEGs related to cancer bone metastasis. (a) Clustered heat map of 1555 DEGs in GSE137842. Red: significantly upregulated genes; blue: significantly downregulated genes. (b) Differentially expressed volcano plots in GSE137842. Red dots: significantly upregulated; green dots: significantly downregulated; and black dots: no significant differences. (c) Clustered heat map of 833 DEGs in GSE32269. Red: significantly upregulated genes; blue: significantly downregulated genes. (d) Differentially expressed volcano plots in GSE32269. Red dots: significantly upregulated; green dots: significantly downregulated; and black dots: no significant differences. (e) Clustered heat map of 88 DE-miRNAs in GSE26964. Red: upregulated genes; blue: downregulated genes. (f) Differentially expressed volcano plots in GSE26964. Red dots: significantly upregulated; green dots: significantly downregulated; and black dots: no significant differences. (g) The common DEGs from GSE32269 and GSE137842 involved in prostate cancer bone metastasis and breast cancer bone metastasis by Venny 2.1.0. (h) List of the common DEGs from GSE32269 and GSE137842.

**Figure 2:** Visualizations of pathway and process enrichment analysis results of DEGs. (a) GO term analysis of DEGs. The vertical axis represents the enrichment score value enriched on the GO term item, and the horizontal axis represents the name of the corresponding GO term item in the GO database. The figure only shows the top 15 terms of each category. BP: biological process; CC: cellular component; MF: molecular function. (b) KEGG enrichment analysis of DEGs. The top 15 clusters with their representative KEGG pathways. The color changes gradually from blue to red, which represents the significant level of enrichment to the pathway, and the redder the color, the greater the significance. The horizontal axis represents the enrichment score of the pathway, the vertical axis represents the corresponding pathway name in the KEGG database, and the size of the circle represents the number of genes enriched in the pathway.

**Figure 3:** The landscape of mRNA–miRNA interactions and PPI networks. (a) mRNA–miRNA interaction network. The graphic visualization uses different shapes representing different gene types: oval represents mRNA, and square represents miRNA. Different colors represent different gene expressions: blue represents downregulated genes, and red represents upregulated genes. (b) Differential expression of MEF2C in bone metastatic and nonbone metastatic prostate and breast cancers. The expression of miR-524-5p in bone metastatic and nonbone metastatic prostate cancer. (c) Protein–protein interaction (PPI) network of DEGs. The globules represent proteins, and the line between the globules represents the interaction between the two proteins.

**Figure 4:** miR-524-5p repressed the proliferation and invasion of DU145 and MCF7 cells. (a) The expression of miR-524-5p in MCF7, DU145, and LNCAP cells. (b) The expression of miR-524-5p was increased in DU145 and MCF7 cells after transfection with miR-524-5p mimics. (c) Inhibition of proliferation of DU145 or MCF7 cells after transfection with miR-524-5p mimics by CCK-8 assay. (d) Inhibition of migration of DU145 or MCF7 cells after transfection with miR-524-5p mimics by transwell assay.

**Figure 5:** miR-524-5p specifically targets MEF2C. (a) The expression of MEF2C in DU145 or MCF7 cells after transfection with miR-524-5p mimics. (b) The protein expression of MEF2C in DU145 or MCF7 cells after transfection with miR-524-5p mimics. (c) Schematic representation of the predicted target site for miR-524-5p in MEF2C. (d) Luciferase activity assay in the wild-type or mutant reporter containing MEF2C 3′ UTR (two sites) when transfected with miR-524-5p mimics or NC in 293 T cells.

**Figure 6:** miR-524-5p promoted the metastasis of DU145 or MCF7 cells in an in vitro 3D model. (a) Bone tissue was cocultured with MCF7 or DU145 cells with or without miR-524-5p mimics. (b) The number of MCF7 or DU145 cells adhering to calvarial bone tissue was counted.

**Table 1:** List of primers.

Gene name	Primer sequence
*β*-Actin-F	GGCTGTGCTATCCCTGTACG
*β*-Actin-R	GGCTGTGCTATCCCTGTACG
MEF2C-F	GCACCAACAAGCTGTTCCAG
MEF2C-R	TGTCTGAGTTTGTCCGGCTC
miR-U6-F	CTCGCTTCGGCAGCACA
miR-U6-R	AACGCTTCACGAATTTGCGT
miR-524-5p	CTACAAAGGGAAGCACTTTCTC

## Data Availability

The miRNA microarray data (GSE26964) and mRNA microarray data (GSE137842, GSE32269) used to support the findings of this study have been deposited in the Gene Expression Omnibus (GEO, https://www.ncbi.nlm.nih.gov/geo/) in NCBI.

## Supplementary Materials

Supplementary 1 Table S1: list of upregulated expressed mRNAs in breast cancer bone metastasis samples from the GSE137842 dataset.

Supplementary 2 Table S2: list of downregulated expressed mRNAs in breast cancer bone metastasis samples from the GSE137842 dataset.

Supplementary 3 Table S3: list of upregulated expressed mRNAs in prostate cancer bone metastasis samples from the GSE32269 dataset.

Supplementary 4 Table S4: list of downregulated expressed mRNAs in prostate cancer bone metastasis samples from the GSE32269 dataset.

Supplementary 5 Table S5: list of upregulated expressed miRNAs in prostate cancer bone metastatic samples from the GSE26964 dataset.

Supplementary 6 Table S6: list of downregulated expressed miRNAs in prostate cancer bone metastatic samples from the GSE26964 dataset.
